# Analysis of KRAS Mutation Status Prediction Model for Colorectal Cancer Based on Medical Imaging

**DOI:** 10.1155/2021/3953442

**Published:** 2021-12-22

**Authors:** Zhen Ren, Jin Che, Xiao Wei Wu, Jun Xia

**Affiliations:** ^1^Department of Gastroenterology, Hanyang Hospital Affiliated to Wuhan University of Science and Technology, Wuhan, Hubei 430050, China; ^2^Department of Combination of Chinese and Western Medicine the Third Hospital of Wuhan City, Wuhan, Hubei 430060, China

## Abstract

This study retrospectively included some patients with colorectal cancer diagnosed by histopathology, to explore the feasibility of CT medical image texture analysis in predicting KRAS gene mutations in patients with colorectal cancer. Before any surgical procedure, all patients received an enhanced CT scan of the abdomen and pelvis, as well as genetic testing. To define patient groups, divide all patients into test and validation sets based on the order of patient enrollment. A radiologist took a look at the plain axial CT image of the tumor, as well as the portal vein CT image, at the corresponding level. The physician points the computer's cursor to the relevant area in the image, and TexRAD software programs together texture parameters based on various spatial scale factors, also known as total mean, total variance, statistical entropy, overall total average, mean total, positive mean, skewness value, kurtosis value, and general skewness. Using the same method again two weeks later, the observer and another physician measured the image of each patient again to see if the method was consistent between observers. With regard to clinical information, the KRAS gene mutation group and the wild group of participants in the test set and validation set each had values for the texture parameter. In a study of patients with colorectal cancer, the results demonstrated that CT texture parameters were correlated with the presence of the KRAS gene mutation. The best CT prediction model includes the values of the medium texture image's slope and the other CT fine texture image's value of entropy, the medium texture image's slope and kurtosis, and the medium texture image's mean and the other CT fine texture image's value of entropy. Regardless of the training set or the validation set, patients with and without KRAS gene mutations did not differ significantly in clinical characteristics. This method can be used to identify mutations in the KRAS gene in patients with colorectal cancer, making it practical to implement CT medical image texture analysis technology for that purpose.

## 1. Introduction

The incidence and mortality rates for colon cancer are ranked fourth and second in the world as shown in Figure 1, respectively. Colorectal cancer is believed to originate from polyps and then progresses to cancer. Also, colorectal cancer also develops through a number of protooncogenes and tumor suppressor genes that mutate together. A total of approximately 4004 people with colorectal cancer will have mutations in the KRAS gene. Early detection and prompt treatment increase the chance of surviving a colon cancer. In advanced colorectal cancer, the primary cause of death is postoperative recurrence and distant metastasis. Therefore, finding better treatments to extend the survival period of patients is critical [1–4].

A monoclonal antibody targeted at EGFR targets its signal transduction pathway. Cetuximab, a monoclonal antibody, has seen widespread use in the treatment of patients with metastatic colorectal cancer in the last few years. Neoadjuvant chemotherapy (prechemotherapy), coupled with molecular targeted drug therapy, was proven in scientific studies to improve the quality of life and survival rate of patients with colorectal KRAS gene wild-type cancer. KRAF testing is recommended for all patients with suspected or proven metastatic colorectal cancer since the 2016 release of the NCCN guidelines. Assessing whether patients with colorectal cancer are suitable for treatment with molecularly targeted drugs depends on determining the status of the KRAS gene [5–11].

The gold standard in the clinic for determining the colorectal cancer gene status is histopathological methods. However, this approach is invasive, and samples from the tumor may be altered due to intratumoral heterogeneity, which could yield different results regarding the nature of the tumor, such as whether it is hypoxic or harboring genetic mutations. Because of these facts, it is imperative to devise a noninvasive, reproducible, and homogenous method to measure gene expression in a tumor because it will reflect the heterogeneity of the tumor [12–15].

Due to their common use in colorectal cancer diagnosis, evaluation of treatment response, and clinical follow-up, CT imaging tests are widely utilized in these settings. Use of postprocessing image processing techniques, such as TA, allows imaging technologies to capture details of tumor tissue that cannot be seen with the naked eye. In contrast, little research has connected CT texture analysis (CTTA) and KRAS gene expression in patients with colorectal cancer. Thus, the goal of our research is to see if CT texture analysis can identify patients with or without KRAS gene mutations, the two key KRAS mutation signatures [16–18].

The contribution of this article can be summarized as follows. This study proves that CT texture analysis technology can be used as an auxiliary method to detect the mutation status of KRAS gene in colorectal cancer. The best diagnostic performance model includes 6 texture feature values of plain scan and enhanced CT images. Using this model to predict the KRAS gene mutation has high diagnostic accuracy, sensitivity, and specificity. Based on this, CT texture analysis technology should be promoted and popularized in clinical practice in order to be used as a preliminary screening method for colorectal cancer patients for KRAS gene mutations.

## 2. Related Work

There were three main methods for obtaining texture parameters, namely, statistical, structural, and model [19]. Among them, the statistical type was a commonly used medical image, which is to extract specific parameter values by using different methods to analyze the gray distribution characteristics of a single pixel and its neighboring pixels, mainly including gray histogram analysis method, gray degree cooccurrence matrix method, and neighborhood gray difference matrix method [20]. Among them, the gray-level histogram analysis method represented the distribution of pixel gray levels in the image and could generate first-order texture features such as mean, variance, skewness, kurtosis, and energy value. The second-order texture features were generated by the gray-level cooccurrence matrix method, which described the distribution relationship between adjacent pixels and could generate texture parameter values such as contrast, uniformity, entropy, and homogeneity. High-level texture features such as roughness were determined by the neighborhood gray degree difference matrix method that is produced, which mainly described the spatial distribution between three or more pixels [21]. Structure type refers to the use of different mathematical morphological methods to process and analyze the structure of the image and to obtain texture features from it, which was suitable for describing more regular texture images. This method was computationally intensive and is mainly used to study the texture characteristics of a specific area [22].

Texture analysis technology had also been used many times in CT and PET-CT images to predict the efficacy of neoadjuvant radiotherapy and chemotherapy for colorectal cancer. Caruso and his team [23] found that five texture parameter values including energy value, contrast, and correlation can be used as imaging markers for predicting the sensitivity of colorectal cancer patients to neoadjuvant chemoradiation. Chee et al. [24] confirmed that in patients with locally advanced rectal cancer who had a better response to nCRT treatment, the lower the entropy value presented by the CT texture image, the higher the uniformity. When using PET-CT combined with texture parameters to study the effect of neoadjuvant radiotherapy and chemotherapy for locally advanced rectal cancer [25], it was found that the higher the ratio of the preoperative standard deviation to the average value, the better the neoadjuvant treatment effect.

Texture analysis technology was also widely used to predict the survival rate of colorectal cancer. Initially, Miles et al. [26] found that the uniformity of portal vein images could be used as an independent predictor when comparing liver CT texture images and CT perfusion image parameters to help predict the survival of patients with colorectal cancer. Another scholar [27] studied and analyzed the enhanced CT texture images of the colorectal cancer lesions, and the results showed that the skewness and kurtosis values could predict the 5-year overall survival rate of patients. Different imaging examination methods combined with texture analysis technology could predict the disease-free survival rate of patients with locally advanced rectal cancer. Another texture analysis based on rectal MRI [28] found that kurtosis could be used as an independent predictor of DFS. Lovinfosse et al. [29] used PET-CT image combined with texture analysis to study the survival and prognosis of rectal cancer, and the results suggested that homogeneity and roughness are related to the DFS of locally advanced rectal cancer. The above studies could prove the feasibility of texture analysis in the prognostic analysis of colorectal cancer. In clinical work, suitable inspection methods could be selected according to the needs. With its advantages of simplicity and ease of operation, texture analysis technology provided certain help for the prediction and prognostic evaluation of neoadjuvant radiotherapy and chemotherapy for colorectal cancer. In view of the large amount of unused information and data contained in images [30], in the future, texture analysis technology should be dedicated to supplement and further improve the method of texture feature extraction [31]. And it was expected that under strict experimental conditions, combined with multimodal imaging images, the heterogeneity of tumors could be more accurately quantified [32], which can make reasonable explanations for the histopathological characteristics represented by different texture feature values. Therefore, texture parameters were expected to be used as new bioimaging markers to guide clinical diagnosis and treatment.

## 3. Material and Method

### 3.1. Research Object

The study was approved by the review board of the institution. A total of 92 patients with colorectal cancer confirmed by histopathology who were treated in a tertiary hospital from August 2017 to September 2020 were retrospectively included. All patients received an enhanced CT scan of the abdomen and pelvis before surgery. In addition, all patients enrolled in the group also received genetic testing. Record the clinical characteristics of the enrolled subjects, including age, gender, tumor location, intestinal wall thickness, tumor TNM staging, and histological differentiation. All patients were divided into the following two groups according to the enrollment time sequence: training set (August 2017 to September 2018) and validation set (September 2019 to September 2020).

### 3.2. Scanning Method

All patients used Siemens Somatom Definition Flash CT (Germany) for enhanced CT scan of the abdomen and pelvis before the operation. The patients were placed in a supine position. Before the scan, the abdomen and pelvis were subjected to routine breath-hold positioning, and then, a plain scan of the abdomen and pelvis was performed. Scanning parameters are as follows: tube voltage 120 kVp, pitch 0.9, tube rotation time 0.5 s, Kernel B30f medium smooth, collimator size 128 × 0.6 mm, scanning layer thickness 5 mm, and layer spacing 5 mm. After the plain scan is completed, use a high-pressure syringe to inject 100 mL of the contrast agent Onipex (300 mg/mL, Shanghai General Medical Group, China) through the patient's anterior elbow vein at a rate of 2.5 mL/s. After injection, the contrast is delayed for 60 seconds. Obtain the venous phase scan image of the abdominal and pelvic department. Both plain scan and enhanced CT scan range from the top of the diaphragm to above the symphysis pubis. After the scan, the CT images of all patients are transmitted to the Medical Image Storage and Transmission System (PACS).

### 3.3. Image Processing and Analysis

Without knowing the patient's clinical and pathological information, two radiologists (with 3 and 5 years of experience in abdominal imaging diagnosis) performed independent reading. The plain scan CT image of the largest level of the lesion and the corresponding portal vein CT image were selected, and the two opinions were determined through negotiation. Transfer the selected image to the texture analysis workstation.

Use TexRAD software to analyze the texture of the selected image. TexRAD software uses Gauss-Laplace (LoG) bandpass filtering algorithm to perform selective image processing and then obtains a series of quantitative texture parameter values through gray histogram analysis. The spatial scale factor (SSF) represents the fineness of the filtered and highlighted image features. The filter radius of the subject represents the size of the SSF. The filter radius includes 0, 2, 3, 4, 5, and 6 mm. SSF = 0 means no filtering. SSF = 2 means that after filtering, the texture feature obtained is fine. SSF = 3 ~ 5 means that the obtained texture features are medium after filtering. SSF = 6 means that after filtering, a rough texture feature is obtained. The texture parameter values generated by TexRAD software mainly include average value, standard deviation, entropy value, positive pixel average value, skewness value, and kurtosis value.

Another physician with 1 year of TexRAD experience will delineate a circular region of interest (ROI) in the abnormal thickened area of the intestinal wall in the selected image and ensure that the area of the region of interest delineated is as large as possible. By artificially setting the threshold value, the part with CT value lower than 50 HU in all pixels in the ROI is automatically filtered. After ROI is selected, texture parameter values corresponding to different SSF values will be automatically generated. Record the texture values of all patients' plain scan and enhanced CT images. Two weeks later, the operator and another physician with 2 years of TexRAD experience used the same method to measure the images of all patients again to evaluate the consistency of the method between and within observers.

### 3.4. Statistical Analysis

The chi-square test was used to compare the differences in gender, tumor location, tumor tissue differentiation, and TNM staging between the two groups of patients in the training set and the validation set (KRAS wild-type group and KRAS mutation group). The independent sample *t*-test was used to compare the differences in age and intestinal wall thickness between the two groups. Before constructing the multiple classifier (MFC), draw the receiver operating characteristic curve (ROC) of each texture parameter value and calculate the area under the curve (AUC). At the same time, the Pearson correlation coefficient is used to calculate the correlation between the texture parameters, and the feature value of any two texture parameters with significant correlation with the lower AUC is removed.

Finally, the retained texture features are combined for support vector machine (SVM) modeling. In the training process, tenfold cross-validation is used to test the accuracy of the algorithm and obtain the model with the best diagnostic performance. Use MATLAB R2016a statistical software and machine learning toolbox to estimate the maximum posterior probability (MAP) of SVM on the basis of training set and validation set data. Then, based on the maximum posterior probability value of the prediction model, the ROC curve of the obtained model is further drawn and the corresponding area under the curve is calculated to evaluate the effectiveness of the selected model in predicting the KRAS gene status of patients with colorectal cancer. Use intragroup correlation coefficient (ICC) to calculate interobserver and intraobserver agreement. It is generally believed that an ICC between 0.41 and 0.60 indicates a fair consistency, 0.61 to 0.80 indicates a moderate consistency, and >0.80 indicates a good consistency. *P* < 0.05 indicates that the difference is statistically significant.

## 4. Experiment

In terms of the above-mentioned clinical characteristics (age, tumor location, intestinal wall thickness, tumor TNM stage, and histological type), there is no significant difference between the KRAS gene wild-type group and the mutant group in the training set and the validation set, as shown in Table 1. AC is ascending colon. TC is transverse colon. DC is descending colon. SC is sigmoid colon. HD is highly differentiated. MD is moderately differentiated. PD is poorly differentiated.

After screening, 6 texture feature values are finally selected for SVM modeling. They are the skewness value of the medium texture feature produced by plain scan CT, the entropy value of the fine texture feature, the skewness value and kurtosis value of the unfiltered feature, and the kurtosis value and mean value of the medium texture feature produced by enhanced CT. Among the six parameters, the single texture parameter with the best diagnostic performance is derived from the entropy value of the fine texture image generated by enhanced CT. The performance is shown in Table 2.

In terms of texture parameters generated by plain scan CT images, the best diagnostic model includes four parameters, namely, the average value of positive pixels without filtering, the entropy of fine texture features, and the skewness and kurtosis of medium texture features. The area under the curve, accuracy, sensitivity, and specificity of predicting KRAS mutations in the training set were 0.95, 90%, 88%, and 95%, respectively. The corresponding values in the validation set were 0.99, 90%, 86%, and 91%. If only the texture value generated by the enhanced CT image is considered, the model with the highest diagnostic performance also includes four parameters, namely, the kurtosis value of the medium texture feature without filtering, the entropy value of the fine texture feature, and the medium texture. The skewness value of the feature using the model to predict the AUC of the KRAS mutant in the training set is 0.92, the accuracy rate is 88%, the sensitivity is 85%, and the specificity is 94%. The corresponding values in the verification set are 0.97, 87%, 84%, and 100%, as shown in Table 3.

The ROC curves of various texture features are shown in Figures 2–5.

## 5. Discussion

The results of this study show that it is feasible to use CTTA to assess the mutation status of KRAS gene in patients with colorectal cancer. If the texture features generated by plain scan and enhanced CT scan are considered at the same time, whether in the training set or the validation set, the model containing 6 texture parameters shows high accuracy, sensitivity, and specificity for predicting KRAS gene mutations. In the training set, the texture feature model of plain scan CT and the texture feature model of enhanced CT have the same specificity for predicting the KRAS mutation of colorectal cancer, but the texture feature model of plain CT has higher accuracy and sensitivity. However, for the validation set, the texture model of the enhanced CT image shows higher accuracy and specificity.

Since medical imaging examination currently plays an important role in the preoperative diagnosis and postoperative follow-up of patients with colorectal cancer, can imaging methods provide certain help for gene mutations in tumor tissues? At present, the common clinical examination methods, including CT, magnetic resonance imaging (MRI), and positron emission computed tomography (PET-CT) examination results, are all obtained by the naked eye of the diagnosing doctor. The information available in the image includes the CT value of the CT scan, the signal intensity in the MRI image, and the standard uptake value (SUV) of PET-CT, which are relatively limited.

Texture analysis technology is currently a research hotspot in the field of tumor imaging. The biggest highlight is that it uses a special filtering algorithm to filter radius values based on different subjects to generate a series of pixel-based grayscale spatial distributions that cannot be recognized by the human eye. The quantitative texture parameter values include entropy, kurtosis, and skewness. Compared with the traditional inspection method, it can deeply dig the data information of the original image and reflect the characteristics of the lesion more comprehensively and in detail. Many studies have shown that the parameter values obtained by texture analysis can quantify the heterogeneity of tumors caused by hypoxia, neovascularization, and necrosis and can even distinguish different pathological and genetic types of tumor tissues. Through clinical research, many scholars have revealed that CTTA can be used to evaluate the clinical staging, neoadjuvant chemotherapy, and prognosis of colorectal cancer. However, the relationship between CTTA and the KRAS gene mutation status of colorectal cancer patients has not received enough attention. In this study, by combining the image information obtained by plain scan and enhanced CT with texture analysis technology, the obtained prediction model has high accuracy, sensitivity, and specificity and is used to identify the presence or absence of the KRAS gene of the research object mutation.

Prior to this, related studies have confirmed that PET-CT image combined with texture analysis technology can provide certain value for identifying colorectal cancer or rectal cancer patients with or without KRAS gene mutations. However, in their study, the texture feature values extracted from the old F-FDG PET-CT did not provide sufficient evidence to identify RAS mutations in rectal cancer. Although there are very few researches on the relationship between imaging examination and the genetic mutation status of lesions, most of them are dedicated to the realization of 18F-FD6/PET-CT. In clinical practice, CT examination is easier to be accepted by the public than 18F-FDG/PET-CT imaging, because CT examination is more economical and time-saving, and it benefits patients a lot. In our study, the AUC, sensitivity, and specificity of the best predictive model used to diagnose patient gene mutations are higher than the corresponding values in this study, and this method of operation has been proven to be highly repeatable. In addition, the results of the study also showed that the clinical background data of all patients in the group had nothing to do with gene expression, which is consistent with our results. Compared with this multicenter study, although our study lacks more detailed texture feature values and has fewer subjects, the final diagnostic efficiency is higher, and it is worthy of clinical application.

The limitations of this study are as follows. First of all, the enrolled cases are relatively small, and it is a single-center study, which has a certain selection bias. Secondly, the acquired texture parameters are all based on gray histogram analysis, and there are fewer categories. We will add more quantitative texture feature values in the next study. Thirdly, this study only analyzed the texture features of the axial CT image of the largest cross section of the lesion and failed to further model the lesion area in three dimensions to obtain more volume texture information; finally, it failed to distinguish between colon cancer and rectal cancer. The research results are discussed separately. The above is expected to be improved and perfected in the next research.

## 6. Conclusion

In conclusion, this study proves that CT texture analysis technology can be used as an auxiliary method to detect the mutation status of KRAS gene in colorectal cancer. The best diagnostic performance model includes 6 texture feature values of plain scan and enhanced CT images, namely, those produced by plain scan CT: the skewness value of the medium texture feature (SSF 5), the entropy value of the fine texture feature (SSF 2), the skewness and kurtosis value of the unfiltered feature (SSF 0), the medium texture feature (SSF 3), and kurtosis value and mean value. This model was used to predict that the KRAS gene mutation has high diagnostic accuracy, sensitivity, and specificity. Based on this, CT texture analysis technology should be promoted and popularized in clinical practice in order to be used as a preliminary screening method for colorectal cancer patients for KRAS gene mutations.

## Figures and Tables

**Figure 1:** Schematic diagram of colorectal cancer.

**Figure 2:** ROC curve of single feature diagnosis model, entropy value of fine texture feature (SSF 2) generated by enhanced CT image.

**Figure 3:** The ROC curve of the texture feature diagnosis model composed of plain scan and enhanced CT, the skewness value of the medium texture feature (SSF 5) produced by the plain scan CT, the entropy value of the fine texture feature (SSF 2) and the nonfiltered feature (SSF 0) skewness value and kurtosis value, and kurtosis value and mean value of medium texture feature (SSF 3) generated by enhanced CT.

**Figure 4:** The ROC curve of the texture feature diagnosis model generated by plain scan CT, the positive pixel average value without filtering (SSF 0), the entropy of fine texture feature (SSF 2), the skewness of medium texture feature (SSF 3), and kurtosis (SSF 5).

**Figure 5:** Enhance the ROC curve of the texture feature diagnosis model generated by CT, the kurtosis value of the unfiltered case (SSF 0) and the medium texture feature (SSF 3), the entropy value of the fine texture feature (SSF 2), and the medium texture feature (SSF 4) skewness value.

**Table 1:** Clinical characteristics of all patients.

Item	Training set		*P*	Validation set		*P*
	Mutation	Wild		Mutation	Wild	
Age	62.1 ± 11.2	58.4 ± 12.9	0.67	58.0 ± 14.4	59.9 ± 9.8	0.71
Male	10	11	0.28	10	8	0.92
Female	17	13		15	8	
AC	7	8	0.91	12	1	0.08
TC	3	0		1	3	
DC	1	2		0	2	
SC	7	9		4	4	
Rectum	9	8		8	6	
Thickness	16.6 ± 3.3	17.2 ± 3.9	0.58	15.4 ± 3.9	14.2 ± 3.4	0.43
HD	8	3	0.54	5	1	0.91
MD	17	18		15	11	
PD	2	3		5	4	
T1	0	0	0.42	0	0	0.36
T2	3	2		0	0	
T3	11	11		14	10	
T4	12	11		11	6	
N0	5	2	0.37	8	6	0.46
N1	9	12		12	9	
N2	13	10		5	1	
M0	6	9	0.11	8	5	0.95
M1	21	15		17	10	

**Table 2:** Predictive results including texture parameters.

Model	Texture	Training set				Validation set			
		AUC	ACC	SEN	SPE	AUC	ACC	SEN	SPE
1-D	Entropy (SSF2)	0.98	0.91	0.84	0.94	0.94	0.89	0.82	1.00
	Skewness (SSF5)								
	Skewness (SSF0)								
6-D	Entropy (SSF2)	0.93	0.92	0.87	0.93	0.97	0.91	0.85	1.00
	Kurtosis (SSF0)								
	Kurtosis (SSF3)								
	Mean (SSF3)								

**Table 3:** The prediction result of a single texture parameter value.

CT	Texture	Training set				Validation set			
		AUC	ACC	SEN	SPE	AUC	ACC	SEN	SPE
Enhanced CT	Kurtosis (SSF0)	0.92	0.88	0.85	0.94	0.97	0.87	0.84	1.00
	Entropy (SSF2)								
	Kurtosis (SSF3)								
	Skewness (SSF4)								
Plain scan CT	Mean (SSF0)	0.95	0.90	0.88	0.95	0.98	0.90	0.86	0.91
	Entropy (SSF2)								
	Skewness (SSF3)								
	Kurtosis (SSF5)								

## Data Availability

The data underlying the results presented in the study are available within the manuscript.
